The article "Psychological Health Intervention of Rural Art and Cultural Communication of Dihuagu in Nanxian County under the Background of Network" was published in 2022. Journal: J Healthc Eng.

# Psychological Health Intervention of Rural Art and Cultural Communication of Dihuagu in Nanxian County under the Background of Network

**DOI:** 10.1155/2022/7309387

**Published:** 2022-02-08

**Authors:** Jie Liu

**Affiliations:** Academy of Music and Dance, Changsha Normal College, Changsha 410100, China

## Abstract

**Background:**

With the development of the Internet, people are facing greater pressure. People in modern society are facing the threat of mental illness. For people with poor mental health, it is necessary to take an appropriate psychological intervention. Nanxian dihuagu is not only a form of folk dance but also a collection of local people's artistic wisdom. Now, Nanxian dihuagu artists use network media to record it.

**Objective:**

Introduce the cultural connotation and value function of dihuagu dance in Mingnan county.

**Methods:**

In this paper, literature and field survey methods, according to the logical analysis method of dance point of view, a detailed analysis of multiculture, from the perspective of comprehensive academic research methods, explore the value and cultural significance of dance.

**Results:**

The Internet has promoted the exchange of local art and culture, and the effective communication has been formed under the promotion of network media. But the Internet age has also led to some problems, and psychological intervention can effectively improve the psychological problems caused by the network.

**Conclusions:**

In this paper, the research process is not limited to the dance itself, at the same time, starting from the local folk customs, focusing on the analysis of the significance and value function of dance culture, which provides a reference for the development and optimization of folk customs. And through the analysis of Nanxian dihuagu, we can know more about the national culture and promote the development of Chinese national culture.

## 1. Introduction

Nanxian dihuagu is a dance performance art with local ethnic characteristics, which is usually held in the traditional Lantern Festival, Spring Festival, wedding, and funeral. It is formed on the basis of the original folk dance and folk musical instruments while absorbing a variety of cultural arts. This kind of art is not only happy and beautiful in music melody but also natural in dance action and full of rich breath of life and unique artistic style, which is deeply loved by people.

### 1.1. The Origin and Development of Dihuagu in Nanxian County

Nanxian dihuagu is a folk art invented by people who work every day. It is close to people's living conditions. This form of folk song and dance art inherits the living state and shows people's real living state by relying on the body language recorded from generation to generation. The inheritance and development of dihuagu in Nanxian County have experienced more than 200 years, and its development process can be roughly divided into five stages: the enlightenment period of the Jiaqing era of the Qing Dynasty, the prosperity period from the Xianfeng era to the Tongzhi era of the Qing Dynasty, the peak period from the early Republic of China to the postliberation period, the decline period from the Cultural Revolution to the end of the 20th century, and the revival period in the new century.

The article "Psychological Health Intervention of Rural Art and Cultural Communication of Dihuagu in Nanxian County under the Background of Network" was published in 2022. Journal: J Healthc Eng.

### 1.2. Definition of Psychological Intervention

Psychological intervention is based on psychological consultation and cognitive psychology, using social psychology to design the intervention process of mental health problems in detail so as to influence their action level (i.e., using specific methods) and adjust their mental state in order to lead their mental state to the expected target state.

Due to the increasing pressure of people's lives and the influence of various environmental factors, people under the background of the modern network are often affected by some bad emotions, thus damaging their mental health [1]. Timely psychological intervention can help to prevent personal injury caused by excessive action, form correct self-awareness and self-evaluation, promote communication with the outside world, and improve the quality of life of intervention objects. Taking into account the characteristics of the Internet age, in previous studies, due to the lack of expansion of art therapy methods such as Internet new media and apps, people receiving treatment are vulnerable to psychological intervention, and flower drum practitioners can express their ideas more simply.

### 1.3. The Influence of Psychological Intervention on the Dissemination of Rural Art and Culture

Rural art is a form of artistic expression, and people can obtain the required network information in a short time and pass on the network information that psychological interveners want to convey to the intervened objects in a convenient way [2]. Now, there are some preliminary exploratory studies on the application of psychotherapy suggestions on dihuagu. However, the research is usually a one-way psychological intervention method, most of which is to discuss the two-way interaction between the psychological intervener and the object, without a detailed discussion of the application of dihuagu in the psychological intervention [3]. From the perspective of reception aesthetics, artistic creation is a process in which the audience and the author create a horizon according to their own psychological understanding, which requires the interaction between them. They can create the color, action, emotion, and other aspects of spiritual communication in the process of interaction and guide the next iteration of creation. In this process, their mental state is constantly improved.

The article "Psychological Health Intervention of Rural Art and Cultural Communication of Dihuagu in Nanxian County under the Background of Network" was published in 2022. Journal: J Healthc Eng.

The purpose of this study is to make a detailed theoretical analysis of the psychological cognitive characteristics of various groups and design the most suitable interactive psychological intervention method for various groups [4]. Moreover, through the experiment of color, material, form of expression, work content, and psychological intervention effect of qualitative and quantitative analysis, it has certain guiding significance for psychological intervention. On the other hand, the use of interactive gradient has a very practical significance for psychological intervention. It can be directly used in the process of psychological diagnosis, psychological consultation, and psychotherapy to effectively and appropriately support the intervention objects to improve their mental health indicators.

### 1.4. Cultural Communication of Dihuagu in Nanxian County under the Background of Network

As a representative of the traditional dance of the Han nationality in Hunan Province, the dihuagu of Nanxian County has been inherited with vivid performance forms and rich and varied songs, which is a vivid portrayal of the culture of Nanxian County. In Nanxian County, the protection of flower drum can activate the national art, promote the development of national culture, and build a harmonious socialist society [5]. First, the flower drum ecosystem must be protected. In Nanxian County, the living environment of Huagu was combined with the natural environment to establish a complete ecological protection area, which saved Huagu culture and became a park to protect Huagu culture.

Fundamentally speaking, as intangible cultural heritage, Nanhua drum dance reflects the collective life, thoughts, feelings, and cultural spirit of the people in Nanxian County. It is the crystallization of the wisdom and great spirit of the people. The content of its dance performance is a mirror of the human spiritual lifestyle. It inherits a prosperous and unique cultural spiritual home [6]. In different historical periods, it has the most typical regional characteristics and is the continuation of history. It reflects the world outlook and living conditions of the people in Nanxian County, reflects the collective spirit and action mode of the people in this fertile land, and improves people's understanding of vision and lifestyle, so it has high historical value.

Nanxian dihuagu dance is the great spiritual and cultural wealth of Nanxian people, the living fossil of local folk culture, the crystallization of working people's wisdom, and the primitive cultural gene of Southwest China [7]. The protection and development of traditional ecological culture can improve the cultural awareness of the whole society and contribute to the recovery and development of culture, as well as the planning and construction of cultural ecology. This dance reflects the way of thinking, aesthetic, and social development of the Nanxian people and also reflects the unique historical and cultural charm of this area, showing its unique cultural value.

The article "Psychological Health Intervention of Rural Art and Cultural Communication of Dihuagu in Nanxian County under the Background of Network" was published in 2022. Journal: J Healthc Eng.

Nanxian dihuagu dance is a kind of Han nationality dance with distinctive performance and rich songs. It has unique local characteristics, unique dance art style, rich life taste, and deep mass foundation [8]. At the Gutian Meeting in 1929, Comrade Mao Zedong advised the Red Army soldiers to sing “flower drum” and other recreational activities. Exploring, rescuing, and protecting Huagu have played a certain role in promoting national art, inheriting national culture, and building socialist spiritual civilization. The essence of Nanxian dihuagu culture is reflected in Nanxian's history, thoughts, habits, etiquette, education, production, and life. We should organize cultural education, cultivate folk artists of Nanxian dihuagu dance, and do our best to explore, rescue, and protect the ecological culture of dance.

## 2. Methods

### 2.1. Participants

In order to better study the use of new online media in Nanxian County, the author has carried out preparations many times, taking the method of going to the scene in person, going to Nanxian County, conducting surveys on local residents, interviewing key figures, and distributing questionnaires to a large number of residents. Surveys and other methods to obtain a large number of documents required information.

### 2.2. Process

According to statistics, a total of 280 paper questionnaires were distributed, and 270 were recovered. According to statistics, Nanxian villagers posted 506 WeChat messages, including 92 students, 280 migrant workers, 54 migrant workers, 42 fishery professionals, 18 pure farmers, and 20 businessmen. According to the characteristics of the questionnaire, the coverage of this questionnaire is wide enough.

### 2.3. Research Design

The survey is analyzed and implemented from four aspects. First of all, it is necessary to understand the understanding of new online media in Nanxian County and the daily use of new online media. Second, it is necessary to understand the characteristics and hotspots of new media users in the Nanxian network [9]. Third, it is necessary to understand the new media users' understanding of the dissemination of national traditional culture. Fourth, it is necessary to understand the impact of online new media users on national culture.

The article "Psychological Health Intervention of Rural Art and Cultural Communication of Dihuagu in Nanxian County under the Background of Network" was published in 2022. Journal: J Healthc Eng.

### 2.4. Data Analysis

SPSS16.0 and Amos 7.0 software were used for data analysis. First, record the statistical questionnaire data, extract the data, and conduct statistical analysis. Then, according to the results of questionnaire statistics and statistical analysis, exploratory factor analysis and confirmatory factor analysis were used to verify the suitability and reliability of each measurement scale.

## 3. Results

### 3.1. Analysis of the Respondents' Understanding of Dihuagu in Nanxian County

According to Table 1, 96.6% of respondents knew or did understand the traditional culture, while only 3.40% did not know the traditional culture at all. Generally speaking, the respondents have a high understanding of traditional culture, but some people do not fully understand the traditional culture. The results show that the investigation content is comprehensive and reliable, which may reflect the original intention of the investigation.

### 3.2. Descriptive Statistical Analysis on the Dissemination of Rural Art and Culture

When establishing the influencing factor model, the author assumes that the level of the communication process and audience level have a certain impact on the social level and verifies the correlation through the correlation analysis between the influencing factors [10]. Based on SPSS, the author analyzes the relationship among personal level, social level, and communication process level. From the data in Table 2, it can be seen that personal concern is obviously related to other factors except communication ability, and government policy at the social level is significantly related to media technology at the communication process level [11]. The cultural environment at the social level is significantly related to the media technology and communication ability at the communication process level, and the media technology and communication ability at the communication process level at the social level are also significantly related. The results show that there is an obvious correlation among personal level, communication process level, and social level.

### 3.3. Time Distribution of Internet Use among Survey Population

From the questionnaire, it can be seen that a total of 515 people were surveyed. 196 people surf the Internet every day, accounting for 38.74%. 138 people (27.2%) used the Internet frequently. 156 people did not surf the Internet, accounting for 30.83%. 16% of the elderly could not access the Internet. Most of them can use the network independently. Therefore, the new Internet media has played a positive role in the popularization of Nanxian culture. Among them, 180 people use the Internet for 1–3 hours a day, accounting for 35.57%, 120 people for 3–5 hours, accounting for 23.7%, and 112 people for less than 1 hour, accounting for 22.3%. From the data, young people use the Internet for a long time (Table 3).

The article "Psychological Health Intervention of Rural Art and Cultural Communication of Dihuagu in Nanxian County under the Background of Network" was published in 2022. Journal: J Healthc Eng.

### 3.4. Survey and Analysis on the Installation of Network Tools among the Survey Population

With the use of mobile phones at the same time, WeChat, QQ, Weibo, and many other types of software were downloaded. WeChat, in particular, can greatly promote people's lives and bring convenience to the communication between the two. In addition, it is also an indispensable communication software in production and life [12]. Among 446 people, 88.14% used instant software, and 238 and 226 people used social networks and video websites, accounting for 47.04% and 44.66% of the total, respectively. Like TikTok, it is fun and popular, and many young people love it. Because of the fast pace of work, many people in Nanxian love it and help Nanxian culture expand rapidly (As shown in Table 4).

### 3.5. Analysis of the Cognition of the Survey Population to the Spread of Dihuagu Culture in Nanxian County

Of the 506 surveyed, 298 people barely know their own culture, accounting for 58.89%. 162 people know their own culture, especially Jienan county culture, accounting for 32.02%, and only 9.09% of the people do not understand the culture of Nanxian County. More than 90 percent of people know their own culture. Of the 506 respondents, 354 responded to spreading the culture of Nanxian County to other countries through various forms of network, accounting for 69.96% [13]. 152 people said their culture was not broadcast abroad, accounting for 30.04 percent. Therefore, most people like to inherit their own culture, which plays a positive role in the popularization of Nanxian culture. Of the 534, 304 used WeChat and TikTok, accounting for 85.88%, while 50 used BBS to contribute only 14.25%. But WeChat is worth mentioning. Because WeChat can send photos and videos through moments, a large number of users from different cultures have poured in, and WeChat has gradually promoted cultural exchanges. The details are shown in Table 5.

### 3.6. Analysis of the Types of Cultural Transmission of the Investigation Population to the Drum Culture

About using the new media channel of the network to spread Nanxian culture, 354 people know these methods, 294 people know the method of using photos, accounting for 83.05%, and 270 people choose text communication, accounting for 76.27%. A total of 230 people chose video communication, accounting for 63.97%, and 122 people chose audio communication, accounting for 34.46%. Because of the intuitive nature of the photos, the spread is relatively simple and high speed, so the acceptance of netizens and fans is relatively high [14]. The best way to transmit is to use language and photos. The effect is better. There are short videos with images and sounds in the videos. You can also use music, especially wedding pictures. The effect is very beautiful. In the circle of friends, the relevant videos and pictures were made public, which provided great convenience for the popularization of Nanxian culture (as shown in Table 6).

The article "Psychological Health Intervention of Rural Art and Cultural Communication of Dihuagu in Nanxian County under the Background of Network" was published in 2022. Journal: J Healthc Eng.

### 3.7. Analysis of Rural Network Use Problems and Psychological Intervention Needs

According to the survey data, people with network psychological problems mainly use the network to play games and chat to make friends, and the proportion of playing games is the highest, accounting for 80%, and making friends accounts for 14.3%. This shows that people with psychological problems due to the Internet like the entertainment function of the Internet [15]. On the contrary, nonnetwork causes psychological problems. In order to achieve the purpose of learning, people tend to use the network to understand and obtain information. On the other hand, the proportion of people who have psychological problems due to the network and those who do not have psychological problems is very high, which is worthy of attention [16]. As shown in Table 7, playing games ranks first among the people who have psychological problems, which indicates that online games are an important factor causing middle school students' psychological problems on the Internet.

## 4. Discussion

### 4.1. Strengthen the Innovation of Communication Means of Dihuagu Culture in Nanxian County

#### 4.1.1. New Style of Dance Vocabulary of Dihuagu in Nanxian County

Nanxian dihuagu, as a folk dance, can be properly and skillfully disassembled and reconstructed, which can not only enrich the vocabulary of dance but also be theoretically constructed for “poetry and painting.” In the process of adaptation and innovation, we can start from the following points.

First, perform the best combination of actions. On the basis of traditional sports, change the original range of movement, intensity, rhythm development, and innovation [17]. On the basis of not changing the basic rhythm, it produced a new dance vocabulary and expanded along the trend to make it more emotional. For example, you can see the combination of simple step and long step squat.

Secondly, break the fixed mode of thinking, and make the dance more professional and artistic. According to the characteristics of the performers, Nanxian dihuagu designs dance movements, which can give full play to their respective advantages. The props and movements used by various roles of men and women can learn from each other, strengthen the fluency of movements, and enrich the vocabulary of dance [18]. For example, in traditional dance performance, dance can fully demonstrate the lifestyle of modern people. The foot movement is more flexible, adding a specific jump action. When dancing, the movements are relaxed, broad, open, and smooth. In addition, acrobatic movements such as “exploring the sea” and “front bridge” were added to improve dance appreciation and professional awareness [19]. Clowns can change the original dance movements. We can give full play to the talents of the actors and choose some specific skills and movements, such as flying feet, rotating feet, sweeping feet, and turning upside down so as to make the warm atmosphere of the scene further rise and fully show the positive and optimistic spirit of Nanxian people.

The article "Psychological Health Intervention of Rural Art and Cultural Communication of Dihuagu in Nanxian County under the Background of Network" was published in 2022. Journal: J Healthc Eng.

Finally, it can add luster to other arts. The creative ideas, processing means, and action design of dance are very innovative, which is the feeling of the current era, the pulse of the times and the action after the processing of modern dance vocabulary [20]. Today's square dance has caused a national fitness heatwave. It can selectively absorb the popular modern dance, hip-hop dance, and square dance, as well as the dance elements of teenagers, middle-aged, and elderly people. With the feelings of modern people, we can make the rhythm of original dance, combine simple movements and famous popular songs, and combine them closely with the modern life of young people [21]. Mix modern elements to show the charm of new art. In order to let people all over the country and even the world know this art form, we must depend on the original taste of Nanxian Dihua drum dance and get people's attention through a number of innovations.

#### 4.1.2. Clever Use of Dihuagu Props and Lighting in Nanxian County

The use of beautiful dance composition, creating beautiful movements, and strengthening the innovation of small tools are helpful to strengthen the stage art performance of Nanhua drum dance. Compared with the “Er Ren Zhuan” in the northeast, the dance skills of Dihua drum dance in Nanxian are insufficient; that is to say, there are few “unique skills” [22]. Nanxian flower encouragers hope to show excellent skills and stage performance and cannot be satisfied with playing flower fans and other original performance skills. In addition to handkerchiefs, flowers, wine cups, chopsticks, umbrellas, and other small props, we must also maximize the use of a variety of small props. For example, in the handkerchief, the traditional flower fan dance has only one simple “rotation” [23]. You can learn skills from the northeast “Errenzhuan,” such as adding a handkerchief around the shoulder and other physical activities to perform. Because the Nanxian Wai drum can be used as exaggerated dance props, it can expand the space of stage performance, and the dance pictures will become more overlapping.

The article "Psychological Health Intervention of Rural Art and Cultural Communication of Dihuagu in Nanxian County under the Background of Network" was published in 2022. Journal: J Healthc Eng.

Stage design enriches the role of dance, produces artistic concepts, stimulates imagination, and improves the overall charm of dance. For example, the accompaniment of Lang's seeing his sister in Gaopo is composed in accordance with the local folk song Lang's seeing his sister in Gaopo. It is just that the sisters who wash clothes by the river become “sisters who put clothes by the river” [24]. When performing on the stage, using new multimedia technologies such as stage lighting and scenery, the background of the stage becomes the scene of lyrics, which fascinates the audience and directly feels the beautiful feelings.

#### 4.1.3. Innovation of Performance Program of Dihuagu in Nanxian County

At the first Nanxian dihuagu Art Festival, Yiyang Ziyang District Cultural Center's “drag bench” and so on can break Nanxian's traditional dance performance projects. In this program, the movement of dance elements and the traditional Nanxian dihuagu movement are retained, focusing on the details of the interaction between the dancers and the clowns [25]. As a flower drum performance, although the changes of dance modeling are relatively scattered, the movements are consistent with the rhythm of fixed music, and the whole is beautiful, neat, and hierarchical. The clown rolls forward from the bench, mastering somersault and other skills, combining with the characteristics of sports, adding a specific story performance plot, setting special performance skills, making the scene warm and the audience in a high mood, meeting the expression of modern people's emotion, temperament, spirit, and sense of rhythm to the greatest extent, and meeting the aesthetic psychology and needs of modern people [26].

Nanxian dihuagu dance can be transformed into a family comedy stage, creating new scripts and beautiful songs. The traditional dihuagu dance can be integrated into family comedy, and the accompaniment music can be integrated into chorus or Male Solo and female lead singing. Various dance segments, such as group dance and double dance, are added to enhance the artistic charm and stage performance of Nanxian dihuagu dance by using multimedia technologies such as stage space layout, original configuration, stage lighting, and scenery [27].

The article "Psychological Health Intervention of Rural Art and Cultural Communication of Dihuagu in Nanxian County under the Background of Network" was published in 2022. Journal: J Healthc Eng.

All the traditional dance projects of the Nanhua drum in Nanxian County need to be sorted out and maintained. For those that are still preserved, they should be selectively absorbed by all means of criticism and modernization and optimized in combination with modern aesthetics. It can adjust and transform the original music songs and movements and create new dance works [28]. Only in this way can we maintain the original vitality of the dance and inherit the traditional art of the country.

We should comprehensively study the contents and forms of flower drum and folk art in different times, regions, and styles, learn the advantages of others, make up for our own weaknesses, absorb the essence, eliminate the bad content, and optimize and improve them in the largest scope [29]. Although the content has changed, the essence remains unchanged. The function of dihuagu dance in Xinnan county still maintains the excellent characteristics of traditional culture, reflects the cultural connotation of the nation, and can adapt to the modern aesthetic and promote the development of modern culture.

### 4.2. Strengthen the Construction of Network Media Tools and Talent Quality in Rural Art Communication

With the development and application of network, human society takes knowledge and network information as the main resources to participate in the construction of a network information society. In the network information society, the relevant talents of Nanhua drum can not only learn multimedia technology and computer network technology and other professional skills but also face a large number of pieces of network information, know how to effectively obtain and identify network information, process network information, express network information creatively, and send network information [30]. Facing the severe challenges brought by the network information age, it is a new historical mission for modern educators to teach students to acquire, evaluate, and apply network information.

#### 4.2.1. Cultivate Network Information Retrieval Skills of Talents Related to Dihuagu in Nanxian County

Before the emergence of the network, the network information retrieval skills mainly refer to the library information retrieval skills for the relevant talents of Nanxian dihuagu University, but now the network environment contains more important network information retrieval skills. This paper mainly introduces the network information retrieval skills under the network environment.

Network information is very rich in content and form, including politics, economy, sports, entertainment, medical care, education, science, and technology, mainly including color photos, text, audio, and video. Faced with the vast amount of network information, if we do not have the ability to search for network information resources, we will not only be unable to obtain effective network information, but also consume a lot of precious time [31]. Many talents associated with dihuagu in Nanxian originally intended to use the network to obtain learning resources, but in the face of many network connections, they did not know how to choose and finally turned their attention to other pieces of external network information; the loss exceeded the gain. Therefore, for educators, it is particularly important to cultivate talents related to Nanhua drum network information retrieval skills. In the network environment, the forms of network information retrieval include search engine and electronic database. Educators should not only teach students how to use search engines and electronic databases to obtain network information methods and skills but also let students quickly and effectively obtain the necessary network information.

The article "Psychological Health Intervention of Rural Art and Cultural Communication of Dihuagu in Nanxian County under the Background of Network" was published in 2022. Journal: J Healthc Eng.

#### 4.2.2. Cultivate Network Information Evaluation Skills of Talents Related to Dihuagu in Nanxian County

Although the network information on the network is rich but complex, there are also a large number of pieces of unfiltered fake network information and pornographic network information [32]. Educators teach students to evaluate the reliability, appropriateness, and correctness of network information from the collected network information so as to prevent students from indulging in the virtual world. Students need to use critical thinking to evaluate these pieces of network information so as to avoid losing the sense of active participation or forming the character of indifference, isolation and lack of responsibility.

#### 4.2.3. Cultivate Network Information Application Skills of Talents Related to Dihuagu in Nanxian County

The cognitive impairment caused by the Internet has sounded the alarm for educators. Therefore, education should not only let students understand the ability to obtain and evaluate network information but also creatively apply network information. Facing the network information, students cannot use it for their own purposes. Educators must guide students to reorganize the network information and combine the new network information with the original knowledge background. Students can use the network information reasonably and effectively, instead of being subordinate to the network information, and can become masters, so as to creatively construct the network information system owned by students.

In the process of cultivating students' network information literacy ability, educators should not put it in the priority of classroom education but should combine it with daily education. Let students develop excellent network information literacy ability unconsciously. In addition, considering the poor level of network dependence, in order to use and rationalize the network as a tool, the relevant talents of Nanhuagu need to introduce network information literacy education in the freshman year.

The article "Psychological Health Intervention of Rural Art and Cultural Communication of Dihuagu in Nanxian County under the Background of Network" was published in 2022. Journal: J Healthc Eng.

### 4.3. Reduce the Problems in the Process of Network Culture Communication through Psychological Intervention

The implementation of psychological intervention is to analyze the causes of psychological problems and formulate the exercise plan related to the success or failure of intervention. The causes of psychological problems caused by the Internet are quite different, and the people who have psychological problems seek different satisfaction on the Internet. Some people want to seek new stimulation on the Internet, some want to make more friends through the Internet, some want to reflect their own values, and some want to ease the pressure of reality through the Internet. Sports are also very rich and can provide athletes satisfaction, which is not the same. In order to interfere with the psychological problems caused by the Internet, we use the conditional emotional response to intervene, specifically analyze the specific causes caused by psychological problems, suggest the intensity of exercise, and formulate a specific intervention plan. It is suggested that the conditional emotional response intervention method should be used in the temporary improvement of psychological problems caused by the network in Nanxian County, and the necessary and appropriate differential treatment should be carried out.

#### 4.3.1. The Psychological Problems Caused by the Internet Can Be Divided into Mild, Moderate, and Severe Psychological Problems

According to the research results, the intervention effect of a conditional effective response is better than that of moderate network psychological problems for mild network psychological problems. It is suggested that intervention should be carried out at the beginning of the problem. Even if there are no psychological problems, colorful sports activities and games will also be used to enrich students' spare time life. On the other hand, it also reduces the students' time using the Internet and the bad behaviors caused by the psychological problems caused by the Internet.

#### 4.3.2. Suggestions on Adjusting the Psychological Problems of Network Culture Communicators through Psychological Intervention

Considering that the change of action needs a long-term accumulation process, we need to use the conditional emotional response intervention method to improve the psychological problems of talents in the Nanhua drum for a short time. The content of training needs to be adjusted according to the degree, reason, and interest caused by the network.

The article "Psychological Health Intervention of Rural Art and Cultural Communication of Dihuagu in Nanxian County under the Background of Network" was published in 2022. Journal: J Healthc Eng.

Nanxian dihuagu related talents have psychological problems due to network reasons; most of them have serious negative self-knowledge, often think that they cannot do it and give up, considering that they have been used to self-verification, or blame the failure caused by some factors on their own failure, and verify that they cannot do it. In order to temporarily improve the psychological problems caused by the Internet, it is suggested to use the conditional emotional response intervention method, and they can doubt their ability. However, please do not let them have absolutely impossible reasons, and only give them a chance to self-verify.

In the experimental study, if we consider that the subjects may change their physical and mental states due to training or other factors, we need to use the conditional emotional response intervention method to temporarily correct the psychological problems caused by network talents. Grasp the feedback information of the test object at any time, understand the physical and mental state of the test object, and formulate, adjust, and implement a timely, scientific, reasonable, and flexible intervention plan according to the feedback network information of the test object.

Considering the important intervention effect of this experimental study, it is suggested that it is necessary to use the conditional emotional response intervention method to temporarily correct the psychological problems caused by the talent network of dihuagu in Nanxian County. According to the actual situation of different individuals, different periods, and different stages, we should appropriately choose the content and time arrangement of this experimental study.

### 4.4. The Influence of Network New Media on the Dissemination of Rural Art and Culture in Nanxian County

#### 4.4.1. The Network New Media Has Expanded the Dissemination Scope of Nanxian Culture

Nanxian people want to promote fish skin painting and other products, basically through radio and television teaching, not only spending time and labor but also spending a lot of money. As we all know, the advertising price on TV is very high, the economic burden of the people in Nanxian County has increased greatly, the product price has risen, and the sales volume has decreased greatly. Through the new media on the Internet, all problems can be solved simply. In the traditional way of communication, there are also people communicating with each other, but this way of communication has fewer people to understand, less influence, high cost, heavy economic burden, and high product cost. After adding new online media, you only need to take photos and videos through your mobile phone, add appropriate instructions, set up a web page, publish Weibo and WeChat, or use a social network platform, which can be seen by a large number of people. Moreover, the people of Nanxian County can record the life of the people of Nanxian County for the first time, anytime and anywhere, and they can also sell their own products. We all know the importance of smartphones in real life, which can be applied to all aspects of life. Now, people's communication completely depends on mobile phones, which is very convenient. Through QQ and WeChat, it is more convenient for people to communicate with each other and spread network information faster. At the same time, the network can connect the whole world, and the space distance between the whole Earth is reduced. With the help of network technology, network new media is moving towards a higher, faster, and stronger direction. The two combinations combine perfectly. As the popularization speed and scope of network information have been greatly improved, Nanxian County has ushered in a good development opportunity. Therefore, the emergence of new network media provides great convenience for the dissemination of Nanxian culture.

The article "Psychological Health Intervention of Rural Art and Cultural Communication of Dihuagu in Nanxian County under the Background of Network" was published in 2022. Journal: J Healthc Eng.

#### 4.4.2. The Network New Media Has Promoted the Dissemination Speed of Nanxian Culture

The new network media is very convenient, and now, everyone has a mobile phone, no matter when and where all parts of life can be recorded. The Wurigong meeting of Nanxian County will be held in Zhangjiakou. It is a comprehensive meeting, including religious belief, sports performance, clothing display, food feast, national song, and dance. The people of Nanxian County are singing and dancing, very lively. People who are not in Zhangjiakou cannot see it on the spot, but in the new media on the Internet, Nanxian culture lovers can enjoy this grand banquet by forwarding the videos, sounds, and photos of mobile phone videos to the Internet. The audience looked at Nanxian County from different perspectives. The grand event was displayed in an all-round way, achieving a good viewing effect and meeting the strong curiosity of the masses and Nanxian cultural lovers. Spreading to the outside world through the new media on the Internet is not only an important channel but also a window for the outside world to understand Nanxian. Nowadays, many ethnic minorities use the new media on the Internet to introduce their national habits and works of art. It provides an excellent platform for the display of minority culture, the interweaving and collision of various cultures, and the integration and exchange of various cultures. It greatly promotes the exchange and cooperation of national culture and constantly innovates and develops national culture. All these are the benefits of new media on the Internet to cultural development.

The article "Psychological Health Intervention of Rural Art and Cultural Communication of Dihuagu in Nanxian County under the Background of Network" was published in 2022. Journal: J Healthc Eng.

#### 4.4.3. The Network New Media Has Widened the Digital Channel of Cultural Communication in Nanxian County

The so-called digitization means that, with the development of science and technology, computers can convert multiple sound signals, image signals, and other signals into digital signals. Compared with the analog signal, the digital signal has made great progress. It can transform numerous complex network information into binary digital code or data format and process multiple sound and image signals on a computer. Due to the existence of a large number of computer storage devices, it is very important for the digitization of Nanxian culture. This means that the national culture can always record the life of the people in Nanxian County and keep many beautiful things, regardless of regional and time restrictions. At the same time, the Nanxian people's marriage habits and other digital forms can also be promoted. This kind of record not only records the grand wedding on the wedding day but also records the preparations before marriage, including how to worship ancestors and the details of married life. It can record all the things about marriage habits from a complete perspective, and it can be spread on the Internet through video. The masses and Nanxian culture lovers can turn on their computers at any time, and they can find pictures and videos of marriage in Nanxian County without time and place restrictions. Such a media digital platform has created many favorable conditions for the continuous inheritance and rapid popularization of Nanxian culture. On the other hand, this network is widely used to shorten the Earth space distance and can spread information to any place on the Earth.

## 5. Conclusion

The basic conclusion of this study is that the Internet era must inherit excellent local traditional culture. This paper adopts the method of literature analysis and visiting survey, starting from the characteristics of rural art, carries out a detailed analysis of multiculturalism, and discusses the value and cultural significance of dance from the perspective of comprehensive academic research methods. This is not only a requirement of the Internet age but also because the local tradition contains the cultural truth of human existence. The culture of the Internet age is not imagined but produced at historic moments according to local traditions. Culture is not a rootless tree. Local tradition is the root of culture in the Internet age, providing valuable cultural resources for cultural construction and development in the Internet age. In the Internet age, people's cultural behavior is bound to be restricted by traditional culture. In the Internet age, people realize the urgency and importance of inheriting the excellent traditional Chinese culture. It is imperative to build the cultural spirit of the Internet age, and traditional regional culture cannot be fully absorbed. Guided by the materialist dialectics of Marxism and the methodology of seeking truth from facts, we must earnestly study and analyze the excellent cultural essence of local traditions, inherit the reasonable and beneficial culture of local traditions, and improve people's overall cultural level.

The article "Psychological Health Intervention of Rural Art and Cultural Communication of Dihuagu in Nanxian County under the Background of Network" was published in 2022. Journal: J Healthc Eng.

## Figures and Tables

**Table 1:** Statistical results of respondents' understanding of dihuagu in Nanxian County.

The level of understanding of Nanxian dihuagu	Frequency	Percentage	Effective percentage	Cumulative percentage
Know very well	30	11.2	11.2	11.2
Have a certain understanding	228	85.4	85.4	96.6
Do not understand at all	9	3.4	3.4	100.0
Total	267	100.0	100.0	

**Table 2:** Descriptive statistics on the dissemination of rural art and culture.

	Mean value	Standard deviation	N
Interest	3.9	952	267
Government policy	4.03	975	267
Cultural environment	3.23	1.589	267
Network media content	3.61	1.246	267
Network media technology	3.58	1.258	267
Network communication talents	3.57	1.176	267

**Table 3:** Time distribution of the Internet use among survey population.

Category item	Number of people	Proportion (%)
1–3 hours	180	35.57
3–5 hours	120	23.72
Less than 1 hour	112	22.13

**Table 4:** Questionnaire on the installation of Internet tools.

Category item	Number of people	Proportion (%)
Instant software	446	88.14
Social network	238	47.04
Video site	226	44.66

**Table 5:** The cognition of the investigated people on the spread of dihuagu culture in Nanxian County.

Category item	Number of people	Proportion (%)
Barely know	298	58.89
Special understanding	162	32.02
Do not understand	46	9.09

**Table 6:** Communication types of dihuagu culture among the investigated people.

Category item	Number of people	Proportion (%)
Pictures and photos	294	83.05
Text spread	270	76.27
Video dissemination	230	63.97
Audio transmission	122	34.46

**Table 7:** Questionnaire of psychological problems in the process of rural network use.

	There is no need for psychological intervention	Need psychological intervention	x	P
Play online games	85 (16.2%)	28 (80%)		
Audiovisual entertainment	162 (30.8%)	2 (5.7%)		
Chat and make friends	114 (21.7%)	5 (14.3%)	85.286	0
Network information search	98 (18.6%)	0		
Learning and knowledge	67 (12.7%)	0		

The article "Psychological Health Intervention of Rural Art and Cultural Communication of Dihuagu in Nanxian County under the Background of Network" was published in 2022. Journal: J Healthc Eng.

## Data Availability

The datasets used and/or analyzed during the current study are available from the author on reasonable request.
